The article "Recognition of the Possible miRNA-mRNA Controlling Network in Stroke by Bioinformatics Examination" was retracted in 2023. Reasons: signs of a paper mill; compromised peer review; unreliable results or conclusions.

# Recognition of the Possible miRNA-mRNA Controlling Network in Stroke by Bioinformatics Examination

**DOI:** 10.1155/2021/6745282

**Published:** 2021-12-13

**Authors:** Wei Li, Jian Li, Yong Yang

**Affiliations:** ^1^Emergency Department of Benxi Central Hospital, Benxi City, Liaoning Province 117000, China; ^2^Department of Thyroid Head and Neck Surgery, Cancer Hospital of China Medical University, Liaoning Cancer Hospital & Institute, Shenyang City, Liaoning Province 110801, China

## Abstract

**Background:**

Based on the latest research of WHO, it has been revealed that more than 15 million people suffer from stroke every year worldwide. Of these 15 million people, 6 million succumb to death, and 5 million get permanently disabled. This is the prime reason for the substantial economic burden on all parts of the world.

**Methods:**

These data have been obtained from the GEO database, and the GEO2R tool was used to find out the differentially expressed miRNAs (DEMs) between the stroke and normal patients' blood. FunRich and miRNet were considered to find potential upstream transcription factors and downstream target genes of candidate EMRs. Next, we use GO annotation and KEGG pathway enrichment. Target genes were analyzed with the help of the R software. Then, the STRING database and Cytoscape software were used to conduct PPI and DEM-hub gene networks. Finally, GSE58294 was used to estimate the hub gene expressions.

**Results:**

Six DEMs in total were selected out from GSE95204 and GSE117064 datasets. 663 DEMs' target genes were predicted, and NRF1, EGR1, MYC, YY1, E2F1, SP4, and SP1 were predicted as an upstream transcription factor for DEMs' target genes. Target genes of DEMs were primarily augmented in the PI3K-Akt signaling pathway and p53 signaling pathway. The network construction of DEM hygiene is potentially modulated by hsa-miR-3591-5p, hsa-miR-548as-3p, hsa-miR-206, and hsa-miR-4503 hub genes which were found among the top 10 of the hub genes. Among the top 10 hub genes, justification of *CTNNB1*, *PTEN*, *ESR1*, *CCND1*, *KRAS*, *AKT1*, *CCND2*, *CDKN1B*, and *MYCN* was constant with that in the GSE58294 dataset.

**Conclusion:**

In summary, our research first constructs the miRNA-mRNA network in stroke, which probably renders an awakening purview into the pathogenesis and cure of stroke.

## 1. Introduction

The second most common cause of uncertain death around the world is stroke. It is also the primary cause of permanent neurodisability [1, 2]. About 17 million stroke cases occur worldwide each year. Apart from that, a 60% decline in stroke mortality between 1968 and 1996 over 29 years has been observed, and the graph of drop slowed down in the 1990s and started gaining pace in several regions of the country [3, 4]. Stroke patients usually require long-term rehabilitation after the acute phase and need to receive continuous community support and nursing home care [5]. The mechanism of stroke is varied. It is crucial to explore new biomarkers associated with stroke pathogenesis.

MicroRNAs (miRNAs) are 18-25-nucleotide-length noncoding RNA molecules that work as master administrative molecules by authorizing large networks of genes, either by destabilizing mRNA transcripts [6], by inhibiting their shift into proteins [7], or by authorizing methylation status of target genes [8]. Although relatively small in number, miRNAs are believed to authorize most tissue- and cell-specific transcriptomes [8, 9]; they also control specific biological processes, which include mitosis, tissue-specific cell differentiation, and cell death [10], sustaining the pluripotent state of ESCs [11], and they delay neuronal maturation or promote neuronal differentiation [12]. miR-17 has been reported to be significantly elevated in patients with acute stroke compared to controls (patients at vascular risk but without stroke) [13]. miR-210 was decreased in those patients who suffered from ischemic stroke compared to controls [14], and stroke outcome was better in patients with higher miR-210 levels [15]. A study has found that miR-124 expression in the central nervous system is a hundred times more than that in other organs [16]. Besides, miR-124 plays a vital part in several developmental processes during CNS development in terms of adult neurogenesis and neuronal demarcations [17]. A lot of research has revealed that miR-320 is consecutively downregulated in stroke patients. These research studies suggest that the downregulation of this miRNA may contribute to the antiapoptotic process [18, 19].

The inspiration of many research studies on the justification and working maneuver of miRNAs in stroke disease has been carried out; however, little research has been conducted on the role of the miRNA-mRNA regulatory network in stroke disease. In the current study, we screened DEMs in stroke tissues compared with normal tissues by analyzing 2 datasets (GSE95204 and GSE117064) from the GEO database for the first time. The transcription factor-DEM, DEM-target gene, functional analysis of target genes, and DEM-hub gene network were performed. In addition, expression levels of hub genes were further verified based on the GSE58294 dataset. Hence, we aimed to construct a potential miRNA-mRNA regulatory network to provide new ideas for diagnosing and treating clinical stroke disease.

## 2. Methods and Materials

### 2.1. Database

To get the gene expression details, 3 Gene Expression Omnibus (GEO) databases (https://www.ncbi.nlm.nih.gov/geo/) were utilized: GSE95204 (miRNA), GSE117064 (miRNA), and GSE58294 (mRNA). The GSE95204 database was based on the GPL18058 platform, GSE117064 was based on the GPL21263platform, and GSE58294 was based on the GPL570 platform. Absolute information is shown in the form of Table 1.

### 2.2. Screening Differentially Expressed miRNAs (DEMs)

GEO2R (http://www.ncbi.nlm.nih.gov/geo/geo2r/) is an aspiring web tool. It allows the users to compare two or more groups of samples in a GEO series. It helps in the identification of genes that are differentially expressed in other conditions of the experiments. We used GEO2R to analyze differentially expressed mRNAs between the normal and stroke patients' blood from GSE95204 and GSE117064 databases. Adjusted *P* value < 0.05 and ∣Log fold change (FC) | >1 were identified as the starting point of DEMs.

### 2.3. Screening Upstream Transcription Factors for DEMs

FunRich (functional enrichment, http://www.funrich.org/) is one of the prior stand-alone software tools. It is used for functional enrichment as well as interaction network analysis of genes and proteins. Based on FunRich, we determined possible upstream transcription factors for DEMs. Adjusted *P* value < 0.05 was considered statistically prominent.

### 2.4. Predicting Downstream Targets of DEMs

miRNet (https://www.mirnet.ca/) is an online instrument that can analyze miRNA and RNA interchange. We used miRNet to predict downstream target genes of DEMs.

### 2.5. Gene Ontology (GO) and Kyoto Encyclopedia of Genes and Genomes (KEGG) Analyses

GO examination classifies the functionality of genes into three divisions: cellular component (CC), molecular function (MF), and biological process (BP). We used GO analysis to comprehend the unique biological characteristics of transcriptomic and genomic data. The KEGG pathway is reckoned as a bundle of databases that can constitute genomes, drugs, diseases, chemical materials, and biological pathways.

### 2.6. PPI Network

PPI information was derived from the online search tool used to retrieve interacting genes (http://stringdb.org/). Then, we visualized interacting genes via Cytoscape software and used cytoHubba, which is a plugin of Cytoscape. It has rank nodes in a preloaded PPI network. cytoHubba constitutes features through several topological algorithms. The Maximal Clique Centrality (MCC) method was utilized to select hub genes as the optimum 30 nodes of the network of PPI.

### 2.7. Expression Analysis of Hub Genes in the GSE58294 Dataset

The GSE58294 database was obtained from the GEO database. The particular dataset was composed on the GPL570 platform (Affymetrix Human Genome U133 Plus 2.0 Array). Samples of GSE58294 were divided into the normal group and stroke group. We used the dataset to comprehend the articulation level of hub genes between the normal and stroke samples. Adjusted *P* value < 0.05 and ∣Log fold change (FC) | >1 were identified as the initiation point of differentially expressed genes (DEGs).

### 2.8. Statistical Analyses

All of the measurement data were performed with SPSS 19.0 statistical software. Student's *t*-test and one-way ANOVA were used to compare the means of two or more groups. The Cox proportional-hazards model was used for multivariate analyses.

## 3. Results

### 3.1. DEMs Were Selected Out from GSE95204 and GSE117064 Databases

GSE95204 and GSE117064 datasets were obtained from the GEO database. Adjusted *P* value < 0.05 and ∣Log fold change (FC) | >1 were identified as the portal of DEMs. 13 DEMs were selected out of the GSE95204 dataset (Figure 1(a)). 823 DEMs were selected out of the GSE117064 dataset (Figure 1(b)). Among all DEMs, we found that 6 DEMs (hsa-miR-548as-3p, hsa-miR-4503, hsa-miR-5194, hsa-miR-3591-5p, hsa-miR-206, and hsa-miR-3127-5p) were consistently changed in both datasets. These results were visualized by using Venn diagrams (Figure 1(c)).

### 3.2. Prediction of Earmark Genes of DEMs and Upstream Arrangement Factors of DEMs' Target Genes

To further determine the role of DEMs between the stroke and normal tissues, we have taken into consideration the FunRich software to predict potential target genes of DEMs. The quantization of target genes for each DEM is listed in Table 2. The DEMs with their target genes were displayed in the DEMs' earmark gene network for better visualization, as shown in Figure 2(a). Transcription factors can bind to mRNAs and exert posttranscriptional regulatory functions, both of which are essential components in the regulatory network in living organisms. FunRich software was utilized to comprehend upstream transcription factors of DEMs' target genes. The results showed 7 upstream transcription factors of DEMs' target genes (NRF1, EGR1, MYC, YY1, E2F1, SP4, and SP1), as shown in Figure 2(b).

### 3.3. GO and KEGG Examinations of DEMs' Earmark Genes

Furthermore, we conducted GO and KEGG examinations on the 663 selected genes of DEMs. We set adjusted *P* value < 0.05 and ranked by *q* value size, selecting the top 10 enrichment features for presentation. BP includes regulation of calcium ion transport, cellular reaction to peptide hormone stimulus, negative regulation of muscle organ development, positive controllability of cyclin-dependent protein serine/threonine kinase activity, postsynaptic density organization, opposite regulation of calcium ion transport into cytosol, supervision of mitochondrial membrane permeability, supervision of smooth muscle cell proliferation, body fluid secretion, and cell death in response to oxidative stress (Figure 3(a)); CC includes cell leading edge, focal adhesion, cell-substrate adherens junction, cell-substrate junction, nuclear chromatin, lamellipodium, ruffle, filopodium, cell cortex part, and sarcoplasmic reticulum (Figure 3(b)); MF includes protein serine/threonine phosphatase activity, histone deacetylase binding, and DNA-binding transcription activator activity, RNA polymerase II-specific (Figure 3(c)); KEGG includes proteoglycans in cancer, prostate cancer, AGE-RAGE beckoning pathway in the case of diabetic issues, PI3K-Akt signaling ways, endocrine resistance, p53 motioning pathway, glioma, fluid shear stress and atherosclerosis, EGFR tyrosine kinase inhibitor resistance, and breast cancer (Figure 3(d)).

### 3.4. DEMs' Target Genes' PPI Network and miRNA-Hub Gene Network of DEMs

The STRING database established DEMs' target genes; Cytoscape software has been utilized to visualize the PPI matrix, and the prior 30 hub genes for DEMs are represented in Figure 4(a). The top 10 hub genes are shown in Table 3: *CTNNB1*, *PTEN*, *ESR1*, *CCND1*, *KRAS*, *AKT1*, *CCND2*, *CDKN1B*, *MYCN*, and *VEGFA*. To better demonstrate the mechanism of DEMs, we conducted a miRNA-mRNA network based on the top 10 hub genes (Figure 4(b)). Results showed that *CTNNB1* and *CDKN1B* are regulated by hsa-miR-3591-5p; hsa-miR-548as-3p regulates *PTEN*; *ESR1*, *CCND1*, *KRAS*, *AKT1*, *CCND2*, and *VEGFA* are regulated by hsa-miR-206; *MYCN* is regulated by hsa-miR-4503.

### 3.5. Hub Gene Articulation Level in the GSE58294 Database

To further determine the role of DEMs in stroke, we used the GSE58294 database to demonstrate the expression level of the top 10 hub genes (*CTNNB1*, *PTEN*, *ESR1*, *CCND1*, *KRAS*, *AKT1*, *CCND2*, *CDKN1B*, *MYCN*, and *VEGFA*) in stroke tissues and normal tissues. Results showed that expression levels of *CTNNB1*, *PTEN*, *KRAS*, *CCND2*, *CCKN1B*, and *MYCN* in stroke tissues are significantly higher compared with those in normal tissues (Figures 5(a)–5(f)). *ESR1*, *CCND1*, and *AKT1* expression levels in stroke tissues are significantly lower than those in normal tissues (Figures 5(g)–5(i)). Only the *VEGFA* expression level was not significantly changed between the normal and stroke tissues (Figure 5(j)). The 9 modified genes are regulated by hsa-miR-3591-5p, hsa-miR-548as-3p, hsa-miR-206, and hsa-miR-4503. Therefore, the menus can serve as potential regulatory pathways in stroke disease.

## 4. Discussion

Stroke remains to be a leading cause of permanent disability. Although stroke mortality has declined over the past 10 years, it is one of the primary causes of death, at number five [20]. Further increments in studies have revealed that biomarkers play a crucial part in the pathogenesis, prognosis, and treatment of stroke [21–23]. It is a type of noncoding RNA sequence. miRNAs constitute very critical biological regulatory functions in many diseases and have been confirmed to have strong relevance to the pathogenesis of stroke [15–17], while the mechanism of miRNA function is still not appropriately known owing to the limited knowledge and comprehension of stroke pathogens [24].

Based on our current research, data from 2 datasets, namely, GSE95204 and GSE117064, have been obtained to point out DEMs linking stroke and normal tissues (blood). A total 6 DEMs (hsa-miR-4503, hsa-miR-206, hsa-miR-548as-3p, hsa-miR-3127-5p, hsa-miR-5194, and hsa-miR-3591-5p) were identified for further analyses. The hsa-miR-206 level was demonstrated as a biomarker for multiple cancers [25, 26] and correlated with muscle function and disease [27, 28]. hsa-miR-3127-5p was identified as a key gene fundamental apparatus of melanoma [29]. In comparison, there are no related research studies about other DEMs.

Numerous studies have proved that miRNAs were regulated with the help of transcription factors [30, 31]. Following this line of thought, we predicted transcription factors of DEMs. Specificity protein 1 (SP1) and specificity protein 4 (SP4) were expected to be the most prominent in the current research. SP1, a C_2_H_2_-type zinc-finger transcription factor [32], has been determined to be strongly associated with stroke disease. SP1 participated in the antioxidant results of curcumin after stroke [33] and enabled it to give protection to neurons after stroke [34]. SP4 has the remarkable ability to reverse numerous prototypes of conventional inflammatory and neuropathic hypersensitivity [35] and regulate constitutive justification of serine racemase in neurons via the NRF2 signaling pathway [36]. Though there is no reported relation between stroke and SP4, its function on neurons might slightly hint at its role in stroke disease. Oxidative stress-elicited transcription factor Yin Yang 1 (YY1) regulates the antioxidative response with the help of enhancement of NRF2-driven transcriptional activity [37, 38]. In the E2F transcription factor 1 (E2F1) study, E2F1 reduced miR-122 transcription to upregulate SPRY2, which stops the MAPK pathway and signifies neurological obstruction in ischemic stroke [39]. EGR1 has been considered and documented as a stroke disease worldwide; researchers have observed that the ischemia-induced EGR1 statement may amplify brain injury by indemnifying the BDNF statement [40]. Additionally, EGR1 was regulated by miR-199b-3p in ischemic stroke [41]. These results support the value of selected candidate DEMs in the pathogenesis of stroke disease.

KEGG results revealed that DEMs were mainly constituted in the PI3K-Akt motioning pathway and p53 signaling pathway. Resveratrol can activate this pathway to render neuroprotection in stroke [42]. Furthermore, the PI3K-Akt pathway is linked with angiogenesis, oxidative stress, and abidance of mesenchymal stem cells under pathophysiological conditions of ischemia [43]. The protein that suppresses tumors is p53; it is also known for regulating critical cellular processes, including cell cycle arrest, DNA repair, senescence, and apoptosis. It interacts with B cell lymphoma 2 family proteins, thereby activating a mitochondrial apoptotic program with greater efficiency than its activity as an arrangement factor [44].

By making the DEM-hub gene network, we observed that the prior hub genes could be primarily marked by hsa-miR-3591-5p, hsa-miR-548as-3p, hsa-miR-206, and hsa-miR-4503. Among the top 10 hub genes, the expression level of 9 genes (*CTNNB1*, *PTEN*, *KRAS*, *CCND2*, *CCKN1B*, *MYCN*, *ESR1*, *CCND1*, and *AKT1*) showed statistically significant differences between the normal and stroke tissues based on the GSE58294 dataset. *CTNNB1*, *PTEN*, *MYCN*, *ESR1*, and *AKT1* have been proved to be associated with stroke disease [45–49]. Therefore, hsa-miR-3591-5p/*CTNNB1*, hsa-miR-548as-3p/*PTEN*, hsa-miR-4503/*MYCN*, hsa-miR-206/*ESR1*, and hsa-miR-206/*AKT1* can serve as potential signaling pathways regulating stroke disease.

We constructed a miRNA-mRNA network in stroke for the first time, while there are still limitations in our current research. Firstly, the sample size of datasets chosen is not huge enough. It is primarily used for biomarker analysis. Secondly, we only conduct bioinformatics analysis without carrying out experiments when determining the role of DEMs in stroke. Therefore, additional research combined with experimental validations in vivo and in vitro is still required to support our examination.

## 5. Conclusion

We firstly construct a miRNA-mRNA network in stroke and demonstrate the potential signaling pathways (hsa-miR-3591-5p/*CTNNB1*, hsa-miR-548as-3p/*PTEN*, hsa-miR-4503/*MYCN*, hsa-miR-206/*ESR1*, and hsa-miR-206/*AKT1*) regulating pathological mechanisms of stroke. Our findings may play a vital role in future in-depth studies and confiscate the goal of the underlying pathology of those who are suffering or have suffered from stroke.

## Figures and Tables

**Figure 1:** Scanning differentially expressed miRNAs (DEMs). (a) DEMs in GSE95204. (b) DEMs in GSE117064. (c) Venn diagram representing the intersection of DEMs in the 2 datasets (GSE95204 and GSE117064). ∣LogFC | >1 and adjusted *P* value < 0.05 were set at the gateway to screen DEMs.

**Figure 2:** Prediction of possible earmark genes of DEMs and upstream transcription factors of target genes. (a) The miRNA-target gene network for DEMs. (b) Transcription factors of DEMs.

**Figure 3:** GO and KEGG annotation: analysis of the target genes of DEMs. (a) Biological process examination for the earmark genes of DEMs. (b) Cellular component earmark for the selected genes of DEMs. (c) Molecular function examination of the selected genes of DEMs. (d) KEGG examination of the prior genes of DEMs.

**Figure 4:** Hub genes for DEMs in the PPI matrix and miRNA-hub gene regulatory network. (a) PPI matrix of the prior 30 hub genes for DEMs. (b) miRNA-hub gene authorization matrix of the top 10 hub genes.

**Figure 5:** The mRNA articulation level of the top 10 hub genes was determined in the GSE58294 dataset. (a) *CTNNB1*. (b) *PTEN*. (c) *KRAS*. (d) *CCND2*. (e) *CCKN1B*. (f) *MYCN*. (g) *ESR1*. (h) *CCND1*. (i) *AKT1*. (j) *VEGFA*.

**Table 1:** Details of GEO databases.

GEO ID	Platform	Sample	Normal	Stroke	Gene/miRNA
GSE95204	GPL18058	Blood	3	6	miRNA
GSE117064	GPL21263	Blood	1612	173	miRNA
GSE58294	GPL570	Blood	23	69	Gene

**Table 2:** Potential target genes of significantly expressed DEMs.

DEMs	Number
hsa-miR-206	122
hsa-miR-3127-5p	64
hsa-miR-3591-5p	98
hsa-miR-4503	71
hsa-miR-5194	135
hsa-miR-548as-3p	173
Total	663

**Table 3:** Top 10 hub genes of the primarily expressed DEMs in the PPI matrix ranked by MCC.

Gene symbol	Score
CTNNB1	2507803436
PTEN	2507772008
ESR1	2507699535
CCND1	2503667182
KRAS	2491184236
AKT1	2270481565
CCND2	2243139386
CDKN1B	2043921875
MYCN	2008662709
VEGFA	1979211433

## Data Availability

Data supporting the results of the study can be available by emailing the first author or corresponding author.

## Additional Points

*Research Highlights*. This research is the first to conceptualize the function of DEMs selected out from GSE95204 and GSE117064 datasets in stroke disease, its function predicted by GO and KEGG inspection, and their focused hub genes, which were further verified based on the GSE58294 dataset. The construction of the miRNA-mRNA network revealed the potential mechanism in stroke and came up with new insight into the pathology of stroke.
